# Differential modulatory effects of GSK-3β and HDM2 on sorafenib-induced AIF nuclear translocation (programmed necrosis) in melanoma

**DOI:** 10.1186/1476-4598-10-115

**Published:** 2011-09-19

**Authors:** Qingjun Liu, James W Mier, David J Panka

**Affiliations:** 1 Division of Hematology-Oncology, Beth Israel Deaconess Medical Center and Harvard Medical School, Boston, MA, USA; 2 Division of Urology, Beijing Friendship Hospital, Capital Medical University, Beijing, China

**Keywords:** Sorafenib, MI-319, HDM2, p53, GSK-3β, Apoptosis-Inducing Factor (AIF), apoptosis, Bcl-2

## Abstract

**Background:**

GSK-3β phosphorylates numerous substrates that govern cell survival. It phosphorylates p53, for example, and induces its nuclear export, HDM2-dependent ubiquitination, and proteasomal degradation. GSK-3β can either enhance or inhibit programmed cell death, depending on the nature of the pro-apoptotic stimulus. We previously showed that the multikinase inhibitor sorafenib activated GSK-3β and that this activation attenuated the cytotoxic effects of the drug in various BRAF-mutant melanoma cell lines. In this report, we describe the results of studies exploring the effects of GSK-3β on the cytotoxicity and antitumor activity of sorafenib combined with the HDM2 antagonist MI-319.

**Results:**

MI-319 alone increased p53 levels and p53-dependent gene expression in melanoma cells but did not induce programmed cell death. Its cytotoxicity, however, was augmented in some melanoma cell lines by the addition of sorafenib. In responsive cell lines, the MI-319/sorafenib combination induced the disappearance of p53 from the nucleus, the down modulation of Bcl-2 and Bcl-x_L_, the translocation of p53 to the mitochondria and that of AIF to the nuclei. These events were all GSK-3β-dependent in that they were blocked with a GSK-3β shRNA and facilitated in otherwise unresponsive melanoma cell lines by the introduction of a constitutively active form of the kinase (GSK-3β-S9A). These modulatory effects of GSK-3β on the activities of the sorafenib/MI-319 combination were the exact reverse of its effects on the activities of sorafenib alone, which induced the down modulation of Bcl-2 and Bcl-x_L _and the nuclear translocation of AIF only in cells in which GSK-3β activity was either down modulated or constitutively low. In A375 xenografts, the antitumor effects of sorafenib and MI-319 were additive and associated with the down modulation of Bcl-2 and Bcl-x_L_, the nuclear translocation of AIF, and increased suppression of tumor angiogenesis.

**Conclusions:**

Our data demonstrate a complex partnership between GSK-3β and HDM2 in the regulation of p53 function in the nucleus and mitochondria. The data suggest that the ability of sorafenib to activate GSK-3β and alter the intracellular distribution of p53 may be exploitable as an adjunct to agents that prevent the HDM2-dependent degradation of p53 in the treatment of melanoma.

## Background

Glycogen synthase kinase-3β (GSK-3β) is a constitutively active kinase regulated primarily by an inhibitory phosphorylation at Ser^9 ^[1] and activated by endoplasmic reticular (ER) and other forms of cellular stress [2,3]. The enzyme has a variable modulatory effect on the response to apoptotic stimuli in that it can either enhance or suppress apoptosis depending on the nature of the stimulus [4]. GSK-3β activation, for example, generally inhibits apoptosis triggered by the engagement of death receptors [4,5] but enhances the apoptotic response to death signals originating in the mitochondria [4,6]. GSK-3β activates NF- κB [7] and phosphorylates hexokinase II, facilitating its association with VDAC [8] in the outer mitochondrial membrane, both of which would be expected to promote cell survival. On the other hand, it phosphorylates c-myc, β-catenin, and numerous other survival-associated proteins leading to their degradation in the proteasome [9,10], thereby facilitating programmed cell death.

Among the downstream targets of GSK-3β are the tumor suppressor p53 and its negative regulator, the E3 ligase HDM2 [2,3,11]. The interaction between these two proteins is governed largely by the extent to which they are phosphorylated by upstream kinases. The phosphorylation of p53 on any of several serines in its N-terminal region, for example, prevents its interaction with HDM2 and enhances its stability in response to stress such as DNA damage or hypoxia [11-15]. N-terminal phophorylation also enhances the acetylation of p53 by the acetyl transferases p300/CBP and PCAF, which facilitates sequence-specific DNA binding by p53 as well as p53-dependent transcription [16]. JNK, p38, ATM and ATR are among the kinases that phosphorylate p53 in this region and promote its activity [11]. The C-terminal phosphorylation of p53 by GSK-3β at Ser^315 ^and Ser^376^, on the other hand, directs the export of p53 from the nucleus and its subsequent degradation in the proteasome [2,17,18]. GSK-3β also phosphorylates HDM2, enhancing its ability to bind and ubiquitinate p53 [8,19]. It is likely that these destabilizing effects on p53 contribute to the prosurvival agenda of GSK-3β in some circumstances.

p53 mediates cell cycle arrest, senescence, and/or programmed cell death in response to DNA damage, hypoxia, and other cellular stresses [20,21]. Although many of these effects of p53 are attributable to its ability to promote gene expression, several are due to the expression of non-coding RNAs or to transcriptional repression. Although p53 resides primarily in the nucleus, there is a substantial cytosolic pool of p53 that in response to an apoptotic stimulus, translocates to the mitochondria, binds to Bax and Bak directly, and induces programmed cell death in a manner similar to that mediated by certain BH3-only members of the Bcl-2 family (i.e. Bim, tBid, and Puma)[22-28]. This particular function of p53 can trigger the release of cytochrome c from the mitochondria, the activation of caspases, and death through a classical apoptotic mechanism. It can also induce a caspase-independent form of death mediated by the translocation of Apoptosis-Inducing Factor (AIF) from the mitochondria to the nuclei. Once in the nucleus, AIF associates with histone H2AX and recruits nucleases such as CypA or EndoG, resulting in the cleavage of DNA into high molecular weight fragments (i.e. programmed necrosis, necroptosis)[29-31]. Both of these mechanisms of programmed cell death are independent of p53-dependent gene expression.

Recently, several small molecule antagonists of HDM2 have been developed which interfere with the interaction between p53 and HDM2, resulting in enhanced p53 stability. Most of these small molecule inhibitors (e.g. the Nutlins, MI-319, and TDP665759) target HDM2 [32-36] whereas others (e.g. RITA) bind to p53 itself [9,37,38]. Both classes of drug increase p53 levels and p53-dependent gene expression without damaging the genome. In the absence of HDM2 blockade, GSK-3β activation (in response to ER stress, for example) leads to the nuclear export of p53 and its subsequent degradation in the proteasome [2,3]. In the setting of HDM2 blockade, however, the p53 exported from the nucleus in response to GSK-3β activation remains available for translocation to the mitochondria in response to apoptotic signaling. Its pro-apoptotic function in the mitochondria is further enhanced by its physical association with GSK-3β [39]. The ability of HDM2 inhibitors to prevent the degradation of p53 that usually follows its nuclear export and the ability of GSK-3β to facilitate the redistribution and mitochondrial function of p53 suggest that combining an HDM2 antagonist with an agent that activates GSK-3β might be a particularly useful antitumor strategy.

We previously demonstrated a high degree of variability in the extent of GSK-3β-Ser^9 ^phosphorylation among BRAF^V600E ^(+) melanoma cell lines and showed that GSK-3β activity in these cells was increased in response to the multikinase inhibitor sorafenib [40], presumably through an ER stress-dependent mechanism. This GSK-3β activation blocked the down modulation of Bcl-2 and Bcl-x_L _and the nuclear translocation of AIF otherwise induced by sorafenib and limited the toxicity of the drug. In this report, we show that in the presence of the HDM2 antagonist MI-319, sorafenib induces the disappearance of p53 from the nucleus and its translocation to the mitochondria in melanoma cells. Both of these effects are GSK-3β-dependent. Although MI-319 alone is minimally toxic in melanoma cells as a single agent, it amplifies the toxicity of sorafenib. The cell death elicited by the combination of sorafenib and MI-319 can be inhibited by pifithrin-μ, an agent known to selectively block p53 function in the mitochondria without affecting p53-dependent gene expression [41]. We further show that, in contrast to the suppressive effect of GSK-3β on the down modulation of Bcl-2 and Bcl-x_L _and the nuclear translocation of AIF induced by sorafenib alone, the ability of the sorafenib/MI-319 combination to induce these effects requires the participation of GSK-3β.

The nuclear accumulation of p53 induced by MI-319 alone appears to be well-tolerated by melanoma cells both *in vitro *and *in vivo*. The multikinase inhibitor sorafenib has been extensively evaluated in melanoma patients both as a single agent and in combination with chemotherapy with disappointing results [42,43]. Our data suggest that the ability of sorafenib to activate GSK-3β and alter the intracellular redistribution of p53 may be exploitable as an adjunct to HDM2 blockade in the treatment of melanoma.

## Results

### Effects of sorafenib on MI-319-induced cytotoxicity and p53-dependent gene expression

To assess the effect of sorafenib on MI-319-induced cytotoxicity, A375 and SKMEL5 melanoma cells were exposed to various concentrations of MI-319 and sorafenib for 20 hr, stained with PI, and then analyzed for viability by flow cytometry. The interaction between the two drugs was evaluated in two studies. In the first, A375 and SKMEL5 cells were exposed to increasing concentrations of MI-319 in the presence (black bars ■) or absence (white bars □) of 10 μM sorafenib (Figure 1A) and in the second, the cells were exposed to increasing concentrations of sorafenib in the presence (black bars ■) or absence (white bars □) of 10 μM MI-319 (Figure 1B). As shown in Figure 1A, MI-319 had negligible single agent toxicity for A375 cells and only modest toxicity for SKMEL5 cells, even at the highest concentration tested (20 μM). However, in the presence of 10 μM sorafenib, MI-319 induced a concentration-dependent increase in PI staining in A375 cells (p < 0.0003, < 0.0023, and < 0.0023 for the drug combination vs. 20 μM MI-319 alone, 10 μM sorafenib alone, and 20 μM sorafenib alone, respectively). SKMEL5 cells were much more sensitive than A375 cells to single agent sorafenib but were unaffected by single agent MI-319. Furthermore, the toxicity of sorafenib in these cells was not appreciably augmented by the addition of MI-319. As shown in Figure 1B, the toxicity of single agent sorafenib was concentration-dependent for both cell lines and in the case of A375 cells, augmented by 10 μM MI-319. MI-319 had no such enhancing effect on the toxicity of sorafenib in SKMEL5 cells.

**Figure 1:** **(A and B)**. Induction of apoptosis in A375 and SKMEL5 cell lines treated with (A) variable concentrations of MI-319 with (black bars) or without (white bars □) 10 μM sorafenib or with (B) variable concentrations of sorafenib with (black bars) or without (white bars □) 20 μM MI-319. Data are presented as the percentage of total cells staining positive for propidium iodide. (**C and D)**. p53 and p21^waf ^levels in A375 and SKMEL5 cell lines treated with **(C) **variable concentrations of MI-319 with or without 10 μM sorafenib or with **(D) **variable concentrations of sorafenib with or without 20 μM MI-319. **(E)**. p53-luciferase reporter activity in transfected A375 and SKMEL5 cells treated with 10 μM sorafenib (S) and/or 20 μM MI-319 (M) for 6 hours. Data are presented as fold increase relative to the activity in the untreated control cells.

To assess the effects of sorafenib on MI-319-induced p53 accumulation and p53-dependent gene expression, A375 and SKMEL5 cells were exposed to increasing concentrations of MI-319 in the presence or absence of sorafenib. As shown in Figure 1C, MI-319 increased p53 levels in A375 and SKMEL5 melanoma cells in a concentration-dependent manner. The expression of the cdk inhibitor p21^waf ^was also induced by the drug. The addition of sorafenib (10 μM) partially inhibited the increase in p53 levels induced by MI-319 and almost completely suppressed the expression of p21^waf^. Similar data were obtained in a related experiment in which a fixed concentration of MI-319 (20 μM) was added to varying concentrations of sorafenib. As shown in Figure 1D, 10 μM sorafenib completely inhibited the expression of p21^waf ^induced by MI-319 in both cell lines. To verify that sorafenib was active as a raf kinase inhibitor, the lysates were also probed for pERK. Since p21^waf ^levels can be regulated by ubiquitination and degradation [44,45], we considered the possibility that the observed effects of MI-319 and sorafenib on p21^waf ^levels were due to changes in protein stability rather than p53-dependent gene expression. To more directly assess the ability of sorafenib to antagonize MI-319-induced p53-dependent gene expression, we examined the effects of both drugs on the activity of a p53-luciferase reporter. As shown in Figure 1E, p53 reporter activity was induced by MI-319 (p < 0.0041 and < 0.0048 for A375 and SKMEL5, respectively) and this induction was prevented with sorafenib (p < 0.0060 and < 0.0010 for A375 and SKMEL5, respectively; MI-319 alone vs. the MI-319/sorafenib combination).

To assess the contribution of p53 to the cytotoxic effects induced by sorafenib and MI-319, A375 cells were stably transfected with a tetracycline-inducible p53 shRNA. The transfectants were then treated with doxycycline and evaluated for their susceptibility to MI-319/sorafenib-induced programmed cell death as determined by flow cytometry. As shown in Figure 2A, exposure to doxycycline blocked the induction of p53 and p21^waf ^by MI-319, confirming our hypothesis that the increase in p21^waf ^levels induced by exposure to MI-319 was p53-dependent and not just due to protein stabilization [44,45]. Doxycycline markedly reduced the toxicity of the MI-319/sorafenib combination (p < 0.0271, Figure 2B), indicating that the toxicity of the MI-319/sorafenib combination was at least partly p53-dependent.

**Figure 2:** **The effect of p53 downmodulation on p21^waf ^expression and programmed cell death induced in A375 cells by the combination of 10 μM sorafenib (S) and 20 μM MI-319 (M)**. A375 cells expressing a tetracycline-regulable p53 shRNA were treated with 3 μM doxycycline overnight and then with sorafenib and MI-319 for 6 hr for the western blots shown in **(A) **or 24 hours for the cell death assays shown in **(B)**. Cell death data are presented as the percentage of total cells staining positive for propidium iodide.

### Effects of sorafenib on the intracellular distribution of p53: Role of GSK-3β

To determine if the dissociation between p53 levels and p53-dependent gene expression observed in cells exposed to sorafenib might be due to a change in the intracellular distribution of p53, A375 and SKMEL5 cells were exposed to MI-319 and sorafenib, lysed, and the lysates fractionated as described in Methods into nuclear and mitochondrial fractions. Cox-4 and c-myc were used as markers to assess the purity of the mitochondrial and nuclear fractions, respectively. As shown in Figure 3A, exposure to MI-319 markedly increased the amount of p53 present in the nucleus of both SKMEL5 and A375 cells. The addition of sorafenib, however, prevented this increase in nuclear p53 and induced the accumulation of p53 in the mitochondria in A375, but not SKMEL5 cells.

**Figure 3:** **The role of GSK-3β in the redistribution of p53 induced by sorafenib in the setting of HDM2 blockade**. **(A)**. Nuclear and mitochondrial p53 levels in A375 and SKMEL5 cells treated with 10 μM sorafenib (S) and/or 20 μM MI-319 (M). In these studies, c-myc and COX4 were used as markers for the nuclear and mitochondrial subcellular fractions, respectively. **(B). (Upper Panel)**. Nuclear and mitochondrial p53 and AIF levels in A375 cells expressing a tetracycline-regulable GSK-3β shRNA treated with 10 μM sorafenib (S) and/or 20 μM MI-319 (M) with or without doxycycline pretreatment. The downmodulation of GSK-3β in the doxycycline-treated cells was validated by western blot. **(Lower Panel)**. Nuclear and mitochondrial p53 and AIF levels in SKMEL5 and SKMEL5-GSK-3β ^S9A ^cells treated with 10 μM sorafenib and/or 20 μM MI-319. **(C)**. Effect of GSK-3β on the pro-apoptotic effects of single agent sorafenib and the sorafenib/MI-319 combination as determined by flow cytometry. Cell death data are presented as the percentage of total cells staining positive for propidium iodide.

We previously demonstrated that sorafenib activates GSK-3β [40], a kinase that phosphorylates p53 at two sites within its nuclear export sequence and regulates its intracellular distribution [2,3]. The constitutive and sorafenib-enhanced activities of GSK-3β were previously shown to be greater in A375 than in SKMEL5 cells [40]. To assess the role played by GSK-3β in the redistribution of p53 induced by sorafenib in the setting of HDM2 blockade, we stably transfected A375 melanoma cells with a tetracycline-inducible GSK-3β shRNA and SKMEL5 cells with a constitutively active GSK-3β (GSK-3β ^S9A^) and examined the response of the transfectants to MI-319 and sorafenib. As shown in Figure 3B, treatment with MI-319 markedly increased the nuclear pool of p53 in all of the transfectants regardless of their GSK-3β status. In A375 cells, the addition of sorafenib largely abolished this nuclear accumulation of p53 and induced its translocation to the mitochondria. Suppression of GSK-3β by adding doxycycline prevented the redistribution of p53 induced by sorafenib. The results obtained with SKMEL5 were comparable to those generated with the GSK-3β-downmodulated A375 cells and consistent with the previous observation that SKMEL5 cells have lower GSK-3β activity than A375 cells [40]. To further implicate GSK-3β activity as a critical determinant of how sorafenib affects the intracellular distribution of p53, we examined the effects of sorafenib and MI-319 in SKMEL5 cells infected with an adenovirus expressing a constitutively active form of GSK-3β (GSK-3β^S9A^). The expression of the GSK-3β^S9A ^construct was verified in these studies by western blot with an antibody to hemaglutinin (HA). As shown in Figure 3B (lower panel), exposure to MI-319 increased the nuclear pool of p53 in SKMEL5-GSK-3β^S9A ^cells and the addition of sorafenib induced its disappearance from the nucleus and translocation to the mitochondria, similar to what was observed in melanoma cell lines with high constitutive GSK-3β activity such as A375. As mentioned above, sorafenib had no effect on the intracellular distribution of p53 in uninfected SKMEL5 cells. These results indicate that GSK-3β activity determines that effect of sorafenib on the intracellular distribution of p53.

We previously showed that the GSK-3β activation induced by sorafenib exposure was prosurvival in melanoma cells in that either the pharmacologic inhibition or downmodulation of the kinase enhanced sorafenib toxicity [40]. To determine if the activation of GSK-3β had a similar protective role in cells exposed to both sorafenib and MI-319, A375 cells stably transfected with a tetracycline-regulable GSK-3β shRNA were treated with 3 μM doxycycline overnight or left untreated and then exposed to sorafenib and MI-319. The cells were then stained with PI and analyzed for viability by flow cytometry. As shown in Figure 3C, the downmodulation of GSK-3β enhanced the toxicity of single agent sorafenib (as previously reported) but reduced the toxicity of the sorafenib/MI-319 combination (p < 0.0062 for sorafenib/MI-319 with or without doxycycline). These data suggest that the toxicity of this drug combination is due to both the increase in p53 levels induced by MI-319 and its mitochondrial translocation, the latter of which is dependent on the activation of GSK-3β.

### Regulation of sorafenib-induced AIF nuclear translocation by p53 and GSK-3β

We previously demonstrated that sorafenib induced the mitochondrial release and nuclear translocation of AIF in melanoma cells sensitive to the drug (e.g. A2058) and that AIF translocation was responsible for the cytotoxic effects of sorafenib in these cells [46]. AIF translocation could not be induced in the more resistant cell line A375. To better define the roles of GSK-3β and p53 in sorafenib-induced AIF nuclear translocation, nuclear and mitochondrial fractions were prepared from various drug-treated melanoma cells and analyzed by western blot for AIF. As shown in Figure 3B (upper panel), the sorafenib/MI-319 combination (but not sorafenib alone) was able to induce AIF nuclear translocation in A375 cells stably transfected with a tetracycline-regulable GSK-3β shRNA in the absence of doxycycline. This pattern of AIF translocation, however, was completely reversed in the presence of doxycycline (i.e. with GSK-3β down modulated). In the absence of GSK-3β, sorafenib alone (but not the sorafenib/MI-319 combination) induced AIF nuclear translocation. Data obtained with SKMEL5 were similar to those obtained with the GSK-3β-down modulated A375 cells in that sorafenib as a single agent induced AIF nuclear translocation in a setting in which the sorafenib/MI-319 combination appeared unable to do so. The results obtained with the SKMEL5-GSK-3β^S9A ^cells were identical to those obtained with A375 in that the drug combination, but not sorafenib alone, induced the nuclear translocation of AIF. These data are consistent with the ability of GSK-3β activation to reduce the toxicity of single agent sorafenib but to enhance that of the sorafenib/MI-319 combination.

### Role of mitochondrial p53 in MI-319/sorafenib toxicity

To assess the contribution of mitochondrial p53 to the cytotoxicity induced by the sorafenib/MI-319 combination, cells were pretreated with pifithrin-μ (10 uM), an agent that blocks the pro-apoptotic effects of p53 in the mitochondria without affecting its transcriptional activity [41]. As shown in Figure 4A, pifithrin-μ pretreatment reduced the toxicity of the sorafenib/MI-319 combination by approximately half (p < 0.0267) in A375 cells, implicating the mitochondria as the dominant site of action of p53 in cells treated with this drug combination.

**Figure 4:** **Inhibition of the mitochondrial function of p53 with pifithrin-μ diminishes the cytolytic activity of sorafenib/MI-319**. **(A)**. Effect of pifithrin-μ(10 μM) on the apoptotic effects of 10 μM sorafenib (S) and 20 μM MI-319 (M) in A375 cells. Cell death data are presented as the percentage of total cells staining positive for propidium iodide. **(B)**. Effect of pifithrin-μ on the nuclear translocation of AIF induced by the sorafenib/MI-319 combination (but not sorafenib alone). c-myc and COX4 were used as markers for the nuclear and mitochondrial subcellular fractions used in these assays. **(C)**. GSK-3β activity determines whether pifithrin-μ inhibits the cell death induced in melanoma cells by sorafenib and MI-319. **(Left Panel)**. A375 cells expressing the tetracycline-regulable GSK-3β shRNA with and without doxycycline pretreatment were treated with sorafenib and MI-319 in the presence or absence of pifithrin-μ. Cell death data are presented as the percentage of total cells staining positive for propidium iodide. **(Right Panel)**. SKMEL5 and SKMEL5-GSK-3β^S9A ^cells were treated with sorafenib and MI-319 in the presence or absence of pifithrin-μ. Cell death data are presented as the percentage of total cells staining positive for propidium iodide. **(D)**. Effect of MI-319 and sorafenib on PARP cleavage in A375 cells.

To determine if the mitochondrial translocation of p53 was responsible for the nuclear translocation of AIF induced by sorafenib/MI-319, A375 cells were exposed to various combinations of sorafenib and MI-319 in the presence or absence of pifithrin-μ. The cells were then fractionated into nuclear and mitochondrial subsets and analyzed for AIF by western blot. As shown in Figure 4B, single agent sorafenib again failed to induce the nuclear translocation of AIF in A375 cells. The translocation was, however, readily achieved with the sorafenib/MI-319 combination but could be blocked with pifithrin-μ, suggesting that it was mediated by mitochondrial p53. Since the mitochondrial translocation of p53 accounts for much of the toxicity induced by the sorafenib/MI-319 combination and depends on sorafenib-induced GSK-3β activation, we suspected that the suppressive effect of pifithrin-μ on drug-induced cytotoxicity might be similarly GSK-3β dependent. To test this hypothesis, the experiments shown in Figure 4A were repeated in additional melanoma cell lines with variable GSK-3β activity. As shown in Figure 4C, pifithrin-μ reduced the toxicity of the sorafenib/MI-319 combination by approximately half (p < 0.001) in A375 cells stably transfected with a tetracycline-inducible GSK-3β shRNA in the absence of doxycycline, similar to its effects on the parent A375 cell line shown in Figure 4A. Suppression of GSK-3β by the addition of doxycycline, however, nullified this protective effect (Figure 4C). Pifithrin-μ also failed to protect SKMEL5 cells from the proapoptotic effects of sorafenib/MI-319 unless the constitutively low GSK-3 activity of these cells was enhanced by the forced expression of GSK-3β^S9A ^(p < 0.0212). Collectively, these data establish a causal link between the activation of GSK-3β, the mitochondrial translocation of p53, and the toxicity of the sorafenib/MI319 combination.

We previously showed that single agent sorafenib induced the release of cytochrome c but not AIF from the mitochondria of A375 cells. Sorafenib-induced caspase activation (PARP cleavage) was delayed in these cells (evident at only 24 hours) and did not appear to contribute to the lethality of the drug as the cells were not protected by the pancaspase inhibitor ZVAD [46]. The combination of sorafenib with MI-319, on the other hand, readily induced the translocation of AIF within 6 hours, at which point PARP was still undetectable (Figure 4D), suggesting that the early toxicity of this drug combination was caspase-independent.

### Effects of GSK-3β activation and HDM2 blockade on sorafenib-induced Bcl-2 and Bcl-x_L _down modulation

As with Bim, tBid, and Puma, the ability of p53 to bind to and activate Bak and Bax in the mitochondria is limited by the relative abundance of anti-apoptotic Bcl-2 family members [22-28]. We previously showed that single agent sorafenib down modulated Bcl-2 and Bcl-X_L _in cells with low constitutive GSK-3β activity (e.g. SKMEL5), but not in cells with high GSK-3β activity (e.g. A375, SKMEL5-GSK-3β^S9A^)[40]. To determine how GSK-3β might affect the ability of the sorafenib/MI-319 combination to down modulate these anti-apoptotic BCL-2 family members, A375-GSK-3β-shRNA cells were exposed to MI-319 and/or sorafenib and then evaluated for Bcl-2 and Bcl-X_L _expression by western blot. As predicted from our earlier studies with unmodified A375 cells [40], single agent sorafenib failed to reduce Bcl-2 and Bcl-x_L _levels in these A375 transfectants in the absence of doxycycline or in SKMEL5-GSK-3β^S9A ^cells (Figure 5). However, the drug down modulated these proteins in SKMEL5 cells and A375 cells in which GSK-3β expression was suppressed by doxycyline. Exactly the opposite results were obtained from cells treated with the sorafenib/MI-319 combination. The combination, for example, induced the down modulation of Bcl-2 and Bcl-X_L _in A375-GSK-3β-shRNA cells in the absence of doxycycline and in SKMEL5-GSK-3β^S9A ^cells, but not in SKMEL5 or A375 cells in which GSK-3β expression was down modulated. These results are in agreement with the data shown in Figure 3B, which demonstrate a similar dichotomous effect of GSK-3β as an enhancer or inhibitor of AIF nuclear translocation depending on the status of HDM2. The data shown in Figure 5 suggest that the mitochondrial translocation of p53 and the pifithrin-μ-suppressible component of the toxicity of the sorafenib/MI-319 combination are both augmented by the GSK-3β-dependent down modulation of Bcl-2 and Bcl-x_L_. The data also demonstrate a hitherto unknown ability of HDM2 activity to determine how GSK-3β activation (e.g. by sorafenib) affects Bcl-2 and Bcl-x_L _expression.

**Figure 5:** **GSK-3β activity and p53 levels (HDM2 blockade) determine whether sorafenib exposure downmodulates Bcl-2 and Bcl-x_L _in melanoma cells**. **(Left Panel)**. A375 cells stably transfected with a tetracycline-inducible GSK-3β shRNA were first treated with doxycycline (or not) and then exposed to sorafenib and/or MI-319. Cell lysates were then probed for Bcl-2 and Bcl-x_L_. **(Right Panel)**. SKMEL5 and SKMEL5-GSK-3β^S9A ^cells were treated with sorafenib and MI-319 and the cell lysates then probed for Bcl-2 and Bcl-x_L_.

### Effects of MI-319 and sorafenib on A375 xenografts

To determine if the antitumor effects of the sorafenib/MI-319 combination on A375 melanoma cells *in vitro *could be reproduced *in vivo*, A375 melanoma xenografts were established in nude/beige mice and the mice then treated with sorafenib (80 mg/kg) and MI-319 (200 mg/kg) individually and in combination. As shown in Figure 6A, the tumor growth curve from mice treated with MI-319 was nearly identical to that of the control group. Treatment with single agent sorafenib had a modest growth-retarding effect (p < 0.007 for sorafenib vs. control). Treatment with the drug combination, on the other hand, resulted in a marked decrease in tumor growth (p < 0.001 for the drug combination vs. each of the other treatment groups).

**Figure 6:** **Antitumor effects of sorafenib and MI-319 on A375 melanoma xenografts**. **(A)**. Growth curves of A375 xenografts from mice treated with control vehicle (C), sorafenib (S), MI-319 (M), or both drugs (MS). Data is presented as tumor volume relative to tumor volume when treatment started. **(B)**. Western blot analyses of whole tumor lysates prepared from tumors excised on day 21.

To assess the effects of drug treatment on Bcl-2 and Bcl-x_L _levels, tumors from the different treatment groups were excised on day 21 and analyzed by western blot. As shown in Figure 6B, Bcl-x_L _levels appeared to be increased by treatment with either single agent MI-319 or sorafenib. The protein was undetectable, however, in the tumors excised from mice treated with the drug combination. A similar pattern was noted for Bcl-2 except that the baseline levels were lower. Of note, erk phosphorylation was not diminished in the tumors from mice receiving either single agent sorafenib or the sorafenib/MI-319 combination, indicating that the antitumor effect of these agents was not the result of raf inhibition.

To assess the mechanism by which the sorafenib/MI-319 combination impaired tumor growth, tumor tissue sections were examined by H&E staining for necrosis, IHC for proliferation (Ki-67) and microvessel density (CD31), and by TUNEL assay. Routine H&E staining revealed a marked increase in the extent of necrosis in tumors from mice treated with either single agent sorafenib or the drug combination Ki-67 staining and TUNEL assays limited to areas of tumor that were not overtly necrotic revealed no differences among the treatment groups (data not shown). Analysis of microvessel density using antibodies to CD31 showed a statistically significant decrease in vascularity in tumors treated with sorafenib alone relative to controls (p < .024) and an even greater decrease in vascularity in tumors treated with the MI-319/sorafenib combination relative to sorafenib alone (p < .006) (Figures 7A and 7B).

**Figure 7:** **(A) Effect of MI-319 and sorafenib on microvessel density in A375 xenografts**. Tumors were stained with CD31. **A**. A representative tumor section from each treatment group is shown. **(B) **Endothelial cells were quantitated using Image Pro 6.0 software. Each bar graph is representative of 6 tumors. **(C)**. Immunofluorescence microscopic evaluation of p53 (red) in tumor cells from A375 xenografts. Drug treatment was as indicated in the figure. COX4 (green) was used as a mitochondrial marker in this study. **(D)**. Immunofluorescence microscopic evaluation of AIF (red) in tumor cells from A375 xenografts. Drug treatment was as indicated in the figure. **(E)**. Immunofluorescence microscopic evaluation of AIF in tumor cells from A375 xenografts. All colors are shown here (i.e. blue = Hoescht (Bisbenzimide H33342) stain, green = COX4, AIF = red). Drug treatment was as indicated in the figure.

Histologic sections were also subjected to wide field immunofluorescence microscopy to assess the intracellular distribution of p53. As shown in Figure 7C, p53 (red color) was scarcely detectable in the tumor cells from control or sorafenib-treated mice. Treatment with single agent MI-319 resulted in a marked increase in p53, which appeared to be confined primarily to the nuclei. In the tumor cells from mice treated with both MI-319 and sorafenib, however, a substantial amount of p53 was present outside the nucleus (yellow color) in apparent association with COX4 (green color), consistent with mitochondrial translocation.

Immunofluorescence microscopy was also used to assess the effect of treatment on the intracellular distribution of AIF. As shown in Figure 7D (red filter only), AIF was excluded from the nuclei of tumors excised from control mice and those treated with either sorafenib or MI-319. However, AIF was clearly present in the nuclei of tumors from mice that received both drugs. Figure 7E shows the same tissue sections with all colors displayed. As shown, the control and single agent-treated tumors have a prominent yellow to red cytosolic signal that is presumably due to the proximity of AIF (red) to COX4 (green) in the mitochondria. The nuclei (Hoescht stain) appear dark blue in each of the tumor sections except those from the mice treated with the drug combination, in which case the blue color is replaced by violet, indicating AIF nuclear translocation. These data suggest that the antitumor activity of the sorafenib/MI-319 combination may be due to a direct apoptotic effect mediated by the p53-dependent mitochondrial translocation of AIF as well as an additive antiangiogenic effect.

## Discussion

Although the HDM2 antagonist MI-319 failed to induce an increase in PI-staining, AIF nuclear translocation, or any other manifestation of programmed cell death in melanoma cells when used as a single agent, it was markedly toxic in some (e.g. A375), but not all, melanoma cell lines when used in conjunction with the multikinase inhibitor sorafenib. The cytotoxic effect of the MI-319/sorafenib drug combination in responsive melanoma cells appears to depend on p53 acting in the mitochondria, an effect determined primarily by the GSK-3β activity of the cell line. Our data indicate that GSK-3β activity is not only required for the drug combination to induce the mitochondrial translocation of p53 but also the down modulation of Bcl-2 and Bcl-x_L _and the nuclear translocation of AIF. The critical role played by GSK-3β in these events contrasts with the largely inhibitory function of the kinase on these parameters when sorafenib is used as a single agent. In the absence of HDM2 blockade, for example, exposure to sorafenib induced the down modulation of Bcl-2 and Bcl-x_L _and the nuclear translocation of AIF only in cells with low GSK-3β activity.

An alternative way of presenting these data would be point out that sorafenib is able to down modulate Bcl-2 and Bcl-x_L _and induce AIF nuclear translocation in cells with low GSK-3β activity only when HDM2 is functional and that HDM2 blockade inhibits these effects. HDM2 blockade, on the other hand, is essential for sorafenib-induced Bcl-2 and Bcl-x_L _down modulation and AIF nuclear translocation in cells with high constitutive GSK-3β activity.

The basis for these context-dependent effects of HDM2 and GSK-3β on the cytotoxicity of sorafenib is unknown but several potential mechanisms may be operative. The cleavage of AIF from the inner mitochondrial membrane prior to its release, for example, is mediated by calpain and this proteolytic event is enhanced by oxidative modification of AIF by ROS [47]. The generation of ROS is regulated by the transcription factor Nrf2, whose activity is in turn enhanced by an association with p21^waf ^[48]. In cells with low GSK-3β activity, p53 remains largely nuclear and it is therefore conceivable that in these circumstances the increase in p21^waf ^induced by MI-319 limits ROS production and the processing and subsequent release of AIF from the mitochondria.

In cells with high GSK-3β activity, HDM2 blockade enhances the ability of sorafenib to induce AIF nuclear translocation and to down modulate Bcl-2 and Bcl-x_L_. There are several mechanisms by which p53 and GSK-3β could collaborate to achieve this effect. For example, GSK-3β is known to phosphorylate CREB, β-catenin, c-myc, and other transcriptional factors that regulate Bcl-2 and Bcl-x_L _expression [1,4,49,50]. Once phosphorylated by GSK-3β, these transcriptional factors become substrates for p53-regulated E3 ligases such as β-TrCP or FBW7 [51-53] and are polyubiquitinated and degraded in the proteasome. It is therefore possible that GSK-3β and a p53-inducible E3 ligase work in tandem to destabilize these transcription factors, resulting in the reduced expression of Bcl-2 and Bcl-x_L_.

Using drug doses that have been previously reported for other xenograft models (see Materials and Methods), MI-319 as a single agent appears to be completely ineffective at constraining the growth of A375 xenografts and sorafenib has only a modest effect. The two drugs together, however, markedly delay tumor growth. The growth suppression induced by the drug combination is associated with many of the biochemical changes observed *in vitro *in A375 cells including the down modulation of Bcl-2 and Bcl-x_L_, the mitochondrial translocation of p53, and the nuclear translocation of AIF. In addition, the vascularity of xenografts from mice treated with MI-319 and sorafenib was decreased relative to that of mice treated with sorafenib alone, which was in turn decreased relative to controls. Since the reduced vascularity of the sorafenib group was not associated with a demonstrable retardation in tumor growth, it is unclear whether enhanced suppression of angiogenesis resulting from the addition of MI-319 accounts for the superior anti-tumor activity of the combination.

## Conclusions

The multikinase inhibitor sorafenib has been extensively evaluated in melanoma patients both as a single agent and in combination with chemotherapy with disappointing results. Our data suggest that the ability of sorafenib to activate GSK-3β and alter the intracellular redistribution of p53 may be exploitable as an adjunct to HDM2 blockade in the treatment of melanoma. Our data suggest that the high p53 levels inducible in melanoma cells with an HDM2 antagonist may not result in programmed cell death *in vitro *or appreciable tumor regression *in vivo *unless the drug is administered in conjunction with a second agent that can facilitate these GSK-3β-dependent cytotoxic effects. The ability of HDM2 inhibitors to prevent the degradation of p53 that usually follows its nuclear export and the ability of GSK-3β to facilitate the redistribution and mitochondrial function of p53 suggest that combining an HDM2 antagonist with an agent that activates GSK-3β might be a particularly useful antitumor strategy.

## Materials and Methods

### Cell lines and reagents

The human melanoma cell lines A375 and SKMEL5 were obtained from ATCC and maintained in RPMI-1640 medium containing 10% fetal bovine serum (USA Scientific), 2 mM glutamine and 50 μg/ml gentamycin at 37°C in 5 percent CO_2_. The SKMEL5 cells are heterozygous for the constitutively active BRAF^V600E ^mutation [54] while the A375 line is homozygous as determined by sequence analysis. Sorafenib was provided by Bayer Pharmaceuticals, New Haven, CT. The MI-319 was provided by Ascenta Therapeutics (Malvern, PA) and Sanofi-Aventis (Paris, France).

### Western blots

Cells were treated as described in Results and then lysed in Lysis Solution (Cell Signaling) supplemented with sodium fluoride (10 μM, Fisher Scientific, Hampton, NH) and phenylmethylsulfonyl fluoride (100 μg/ml, Sigma-Aldrich, St Louis, MO). Lysates were fractionated in 8-16% gradient SDS-polyacrylamide gels as indicated and the separated proteins were transferred to nitrocellulose. The blots were probed for the proteins of interest with specific antibodies followed by a second antibody-horse radish peroxidase conjugate and then incubated with SuperSignal chemiluminescence substrate (Pierce, Rochford, IL). The blots were then exposed to Kodak X-Omat Blue XB-1 film. The p21, phospho-p53 (Thr^55^), Bcl-x_L _and AIF antibodies were obtained from Santa Cruz Biotechnology (Santa Cruz, CA); the phospho-erk, c-myc, Bcl-2, p53, phospho-p53 (Ser^315^), Bax, HA-tag, PARP and GSK-3β antibodies were purchased from Cell Signaling (Beverly, MA). The Bak antibody was from Calbiochem (San Diego, CA). The vinculin antibody was obtained from Sigma (St. Louis, MO); the COX4 antibody was obtained from ABCAM (Cambridge, MA).

### Cell death assays

In each of these assays, the adherent cells were detached from the underlying plastic by treatment with trypsin/EDTA in PBS for 5 minutes and then combined with the floating, nonadherent cells. Propidium iodide (PI, 5 ng/ml, Sigma) was added to the cell pool and after 20 minutes at room temperature, the cells were analyzed by flow cytometry with a BD Biosciences FACScan. The percentage of cells staining with propidium iodide (PI) was recorded and each experiment reported was carried out at least 3 times. Data were reported as the mean +/- standard error for each experimental condition. In each of these assays, the percentage of cells staining with PI was taken to represent the extent of cell death induced by the experimental condition being tested.

### p53 reporter assay

A p53 reporter vector containing the p53 response element coupled to firefly luciferase was purchased from Stratagene (Agilent Technologies, Santa Clara, CA). Briefly, tumor cell lines were transfected with the p53 luciferase and a CMV renilla luciferase vector (a gift of Stephen Balk, BIDMC) using Superfect (Qiagen) following the manufacturer's protocol. Twenty-four hours later, the cells were treated with sorafenib (10 μM) and MI-319 (20 μM) for 6 hours. The lysates were assayed using the Dual-Luciferase Reporter Assay System from Promega Corporation (Madison, WI). The data are presented as the ratio of firefly to renilla luciferase activity normalized to untreated controls.

### Subcellular fractionations

Mitochondria-enriched and cytosolic fractions were isolated from Dounce-homogenized cells using the ApoAlert Cell Fractionation Kit (BD Clontech). The quality of the mitochondria-enriched fractions was validated by Western blot using an antibody for the mitochondrial protein cytochrome c oxidase subunit IV (COX4) [55]. Cytosolic fractions were obtained during the isolation of the mitochondria. Nuclei were isolated according to a standard protocol [56], lysed, and analyzed by western blot.

### Design and construction of genetically modified melanoma cell lines

The generation of SKMEL5 cells expressing a constitutively active GSK-3β was previously described [40]. To generate the p53 and GSK-3β shRNA transfectants, the shRNA sequence selector and shRNA hairpin oligonucleotide sequence designer software provided by BD Clontech was used to select optimal sequences. Three shRNAs were generated for each gene to be silenced. To produce tetracycline-regulable shRNAs, the oligonucleotides selected were cloned into the pSingle-tTS-shRNA vector (BD Clontech). This vector is a tet-on vector. The three shRNA constructs were transfected as a group into A375 cells and stable transfectants obtained by selection in G418. Clones were screened individually for inducible expression of the shRNA (i.e. the downmodulation of the gene of interest as determined by Western blot) and 2-3 representative clones were selected for each shRNA based on the degree to which tetracycline exposure suppressed the expression of the gene of interest.

### Immunoprecipitation experiments

Immunoprecipitations were carried out using a Protein A Immunoprecipitation Kit purchased from Roche Diagnostics (Mannheim, Germany). Briefly, treated cells were lysed and subjected to Dounce homogenization, followed by a pre-clearing step with protein A-sepharose. The cleared lysates were incubated with 10 μg primary antibody for 3 hours at 4°C, followed by an overnight incubation with protein A-sepharose. After washing with increasingly stringent buffers, the immunoprecipitated proteins were subjected to western blot analysis as described above.

### Xenograft model

All animal studies were conducted according to Animal Investigation Committee (AIC)-approved protocol of Beth Israel Deaconess Medical Center. Six to eight week old athymic nude/beige female mice (Charles River Labs) were implanted subcutaneously with 1.0 × 10^7 ^A375 melanoma cells. When the tumors reached 7-8 mm in diameter, the mice were divided into 4 treatment groups of 6 mice each and treated daily for 21 days by gavage with sorafenib (80 mg/kg), MI-319 (200 mg/kg), sorafenib + MI-319, or saline (control). The doses of sorafenib [57,58] and MI-319 [59,60] were as previously reported. Tumors were measured bidimensionally daily. Tumor tissue from the sacrificed mice was frozen in liquid N_2 _for western blot analysis as described in Results or fixed in formalin for paraffin embedding.

### Immunohistochemistry and immunofluorescence microscopy

The paraffin-embedded tumor tissue was sectioned at 5 microns using a Leica RM 2125 rotary microtome. The sections were dewaxed at 60°C, serially immersed in solutions of decreasing alcohol concentration, and then boiled in 10 mM sodium citrate, pH 6.2, for 30 minutes to unmask antigens. The tissue was then incubated in 3% hydrogen peroxide for 5 minutes, blocked with 1% BSA and 5% goat serum, and incubated overnight at 4°C with an antibody to Ki-67 (Dako, Carpinteria, CA). The Ki-67 epitope was detected using a biotinylated anti-mouse Ig antibody and an avidin-horseradish peroxidase conjugate (Vector Laboratories, Burlingame, CA). Similarly, sections were stained for endothelial cells with an antibody to CD 31 (ABCAM), followed by a biotinylated anti-rabbit Ig antibody (Vector Laboratories, Burlingame, CA). Slides were then counterstained with hematoxylin, dehydrated, and mounted.

The sections were assayed for apoptosis using the TUNEL method (Millipore, Billerica, MA) in accordance with an established protocol [61]. The tissue was hydrated and treated sequentially with proteinase K and hydrogen peroxide, and then blocked as described above for the Ki-67 staining. The sections were then exposed to a solution containing mixed nucleotides, some of which were digoxygenin-labeled, and terminal deoxynucleotidyl transferase (TdT). The slides were developed with an anti-digoxigenin antibody-peroxidase conjugate and DAB substrate. Tissue staining was quantitated using IMAGE Pro 6.0 software (MediaCybernetics, Inc, Bethesda, MD).

Immunofluorescence microscopy was utilized to assess the translocation of p53 and AIF to the nuclei and mitochondria, respectively. For p53, the above protocol for IHC was followed using a COX 4 antibody conjugated to Alexa 488 (green) and a p53 antibody conjugated to Alexa 555 (red) (both from Cell Signaling, Danvers, MA). For AIF staining, a primary AIF rabbit antibody was used (Santa Cruz) followed by a secondary antibody to rabbit IgG conjugated to Alexa 555, along with the COX 4 antibody-Alexa 488 conjugate. Finally, nuclei were stained with Bisbenzimide H33342 (Alexis Biochemicals, San Diego, CA). Immunofluoresence microscopy was carried out with a Nikon TE-2000E microscope at 100X magnification and a Hamamatsu Orca ER camera. The data was acquired with Nikon's NIS-Elements and analyzed with ImageJ software.

### Statistical analysis

*In vitro *data depicted as bar graphs represent mean values from at least 3 separate experiments +/- standard error. For most of the studies shown, the significance of an apparent difference in mean values for any parameter (e.g. the percent of cells staining with propidium iodide) was validated by a Student's unpaired *t *test and the difference considered significant if p < 0.05. For the xenograft studies, the growth curves of the different treatment groups were statistically compared using one-way ANOVA.

## List of abbreviations

AIF: apoptosis inducing factor; GSK: glycogen synthase kinase; ER: endoplasmic reticular; HDM2: human double mutant 2; HA: hemaglutinin.

## Competing interests

The authors declare that they have no competing interests.

## Authors' contributions

QL carried out many of the xenograft experiments, immnuohistochemistry, wide field fluorescence and western blots. JM conceived of the study, and participated in its design and coordination and helped to draft the manuscript. DP also conceived of the study, and participated in its design and coordination and helped to draft the manuscript. In addition, DP performed all in vitro experiments including the generation of tet-regulable shRNA cell lines and their implementation, cell death assays, western blots, reporter assays and cellular fractionations. All authors read and approved the final manuscript.
